The article "Osteogenic ability of bone marrow stem cells intraoperatively enriched by a novel matrix" was published in 2014. Journal: Exp Ther Med.

# Osteogenic ability of bone marrow stem cells intraoperatively enriched by a novel matrix

**DOI:** 10.3892/etm.2014.2067

**Published:** 2014-11-12

**Authors:** QING YE, KAINING CHEN, WU HUANG, YUNSONG HE, MINGSHAN NONG, CHUNXIANG LI, TIANSEN LIANG

**Affiliations:** 1 Department of Orthopedics, The General Hospital of the Armed Police Force of Guangxi, Nanning, Guangxi 530003, P.R. China; 2 Center of Tissue Engineering Research and Application, The General Hospital of the Armed Police Force of Guangxi, Nanning, Guangxi 530003, P.R. China; 3 Department of Neurology, The General Hospital of the Armed Police Force of Guangxi, Nanning, Guangxi 530003, P.R. China

**Keywords:** poly-L-lysine, demineralized bone matrix, bone marrow stem cells, intraoperatively, matrix

## Abstract

Poly-L-lysine (PLL) is commonly used as an adhibiting agent due to its good viscosity, and demineralized bone matrix (DBM) is a common enriched matrix for selective cell retention technology. Therefore, the aim of this study was to use PLL to coat the surface and interspaces of DBM to form a novel type of enriched matrix [DBM coated with PLL (PLL-DBM)], in order to effectively improve the enrichment effects of bone marrow stem cells and enhance their osteogenic ability. Electron microscope scanning and the infrared spectrum were used to observe the structure of PLL-DBM and the optimal conditions for the combination of PLL and DBM. Enriching effects on bone marrow nucleated cells (NCs) and platelets (PLTs) were detected with an automated hematology analyzer. The osteogenesis of the following four groups was assessed with a grafting bone model in a goat spinal transverse process: IA, tissue engineered bone (TEB) fabricated following enrichment of bone marrow with PLL-DBM; IB, autogenous iliac bone; IIC, TEB fabricated following enrichment of bone marrow with DBM; IID, blank DBM. The goats were sacrificed in one batch at week 16 after the surgery and the fusion specimens were examined using X-ray and three-dimensional computed tomography (CT). In addition, the CT value was determined and the histology and biomechanics were analyzed in order to evaluate the osteogenic ability. The results showed that PLL and DBM combined well and that PLL-DBM exhibited a natural mesh pore structure. The fold enrichment of NCs and PLTs with PLL-DBM was significantly higher than that with DBM. The fusion effects of the IA and IB groups were similar and significantly enhanced compared with those of the IIC and IID groups. The results confirmed that PLL-DBM is an ideal enriched matrix for bone marrow stem cells, and TEB rapidly fabricated by PLL-DBM intraoperatively enriched bone marrow stem cells exhibits an improved osteogenic ability.

## Introduction

There is a significant clinical requirement for bone repair material with high osteogenic activity, and there are ~500,000 cases of bone graft operations every year in the USA (1). Rapid construction of tissue engineered bone (TEB) with high osteogenic activity for immediate use upon demand has become a key study area in the TEB field. Previous studies have demonstrated that a large number of osteoblastic progenitors and osteoinductive factors (OIFs) are contained in red bone marrow, including mesenchymal stem cells, which can differentiate into osteoblasts (2); hematopoietic stem cells, which can promote the vascularization of tissue (3); platelets (PLTs), which can secrete bone growth factors (4) and a number of other OIFs. The utilization of those effective components in bone marrow in the repair of bone tissue has gained significant focus in recent years. Certain effects have been achieved in repairing bone and the treatment of nonunion by local marrow injection (5,6); however, the cell concentration is low and the easy loss of cells decreases the osteogenic ability.

Connolly (7) found that the clonality of osteoblastic progenitors could be enhanced when bone marrow was concentrated, and that bone repair materials combined with concentrated bone marrow could enhance its osteogenic potential. Furthermore, this enhancement in osteogenic potential had a proportional correlation with the number of osteogenic cells. Based on these results, Muschler *et al* (8–11) described a novel technology of enriching bone marrow stem cells, known as selective cell retention (SCR) technology. The mechanism of SCR was that, when bone marrow moved through the proper mesh structure of the matrix, bone marrow stem cells and certain OIFs were selectively detained due to good surface adhesion of the matrix; thus, marrow stem cells and OIFs were enriched while few erythrocytes and lymphocytes were detained (10). Muschler *et al* (10,11) successively took allograft cancellous chips and demineralized cortical bone powder as matrices, and utilized SCR technology to increase the fold enrichment of osteoblastic progenitors. Using SCR technology, Brodke *et al* (12) took allogenic bone fiber and demineralized cancellous bone chip mixtures to enrich osteoblastic progenitor cells, and then mixed SCR-enriched grafts with PLT-rich plasma or non-heparinized marrow mass. The authors found similar osteogenic ability to autogenous bone in dog models of femoral defect. Based on these studies and using the CELLECT™ SCR device (Depuy, NY, USA), Lee and Goodman (13) achieved a therapeutic effect in treating secondary osteonecrosis of the femoral condyles using demineralized cancellous bone chip mixtures as the matrix.

However, the matrices used in the aforementioned studies were blank demineralized bone matrices (DBMs) or cancellous bone chips, which were not coated with a surface modifier; therefore, the ideal effect of bone marrow cell enrichment could not be achieved. Furthermore, the core technology of SCR was designed to improve the adhesion properties of matrix material to bone marrow cells. The aim of the present study was to enhance the enriching effect by coating the DBM surface and inner wall of pores with poly-L-lysine (PLL) and therefore provide an ideal PLL-DBM for SCR technology. In addition, although in recent years there have been a number of reports on SCR technology (11,13–17), the use of the lumbar intertransverse goat model has not been reported. Since the space of the lumbar transverse process of the bone graft model is rather wide but the bone bed surface is relatively narrow, repair materials with a superior osteogenic activity are required for bone fusion; the materials with a poor activity undergo absorption, leading to fusion failure. The conditions of the graft bed in this model are similar to those in the human body and it is a common fusion method in clinical trials. Thus, the goat lumbar transverse process was selected as a bone graft model in this experiment, with the aim of verifying whether PLL-DBM exhibits improved osteogenic activity and providing experimental evidence for clinical applications.

## Materials and methods

### Preparation of DBM and PLL-DBM

The proximal ends the of femoral and iliac cancellous bones of 10 healthy adult males goats (offered by the Animal Center of the General Hospital of the Armed Police Force of Guangxi, Nanning, China) were removed without cartilage or cortical bone, and were sectioned into cubes measuring 5×5×5 mm. Bone blocks were obtained from the tissue engineering bone banks of The General Hospital of the Armed Police Force of Guangxi (Nanning, China). The cleansing and disposal of the DBM were in accordance with the standards for humans in clinics published by Maddox *et al* (18).

Under sterile conditions, the prepared DBM was soaked in 0.1% PLL (P1399; 150–300 kDa; Sigma, St. Louis, MO, USA) for 20 h. A previous study showed that 0.1% PLL resulted in an improved adhesion compared with PLL at a lower concentration, while higher concentrations of PLL did not improve adhesion further (19). Adhesion of PLL on bone marrow cells showed a degree of saturability; therefore, 0.1% PLL was selected in this study. The DBM was then suctioned and filtered with vacuum negative pressure for 10 h until no air bubbles appeared, enclosed following cryodesiccation for 48 h in a lyophilizer, sterilized by cobalt-60 irradiation and preserved in a refrigerator at −20°C.

### Scanning electron microscope observation

Hitachi S-3400N scanning electron microscopy (Hitachi High-Technologies Corp., Tokyo, Japan) was used for scanning electron microscope analysis of the DBM and PLL-DBM, and the Labworks™ image analysis system (UVP, Inc., Upland, CA, USA) was used to determine the pore size and porosity.

### Infrared spectrum analysis

Five sections of PLL-DBM or DBM materials from the same donor were sampled randomly and 5 mg PLL was weighed with a balance. All specimens were ground into a powder to prepare samples. To analyze the components of the samples, a Nexus Fourier transform infrared spectrometer (Nicolet™; Natus Medical, Inc., San Carlos, CA, USA) was used to scan between 4,000 and 5,000 cm^−1^.

### Detection of the enrichment effect for bone marrow nucleated cells (NCs) and PLTs

Referring to the method of Muschler *et al* (8), 30 ml heparinized bone marrow (1,000 U/ml) was harvested from the bilateral posterior superior iliac spine of goats under sterile conditions, and fat cells, clots and bone fragments were removed through the 300-μm filter. The sample was oscillated and agitated for use. The internal tube of the CELLECT device (DePuy Spine, Inc., Raynham, MA, USA) was moistened with 1 ml heparin sodium solution on a sterilized table, and then the DBM or PLL-DBM samples were placed in the filter bowl of the CELLECT device subsequent to being weighed. The bone marrow (1 g PLL-DBM:6 ml bone marrow) was subsequently rolled into the bowl following agitation. The spring of the device was pressed manually, and the return of the spring caused negative pressure so that the bone marrow flowed slowly through the PLL-DBM material. The TEB was then fabricated after three circulations, the effluent bone marrow was collected, the TEB was weighed and the bone marrow volume in the TEB (the retention volume) was calculated.

Specimens of original bone marrow and load effluent were collected and fully agitated. While using an automatic blood cell analyzer (Suzhou Purification Equipment Factory, Suzhou, China), the concentrations of NCs and PLTs of the original sample and load effluent were calculated. Referring to the method of Muschler *et al* (11), the calculation formulae were as follows: i) Cell number of original bone marrow = volume of original bone marrow × concentration of original bone marrow; ii) cell number of load effluent = volume of load effluent × concentration of load effluent; iii) cell number in TEB = cell number of original bone marrow − cell number of load effluent; iv) cell concentration in TEB = cell number in TEB/retention volume; v) fold increase in concentration (α) = cell concentration in TEB/cell concentration of original bone marrow. The final formula was utilized to indicate α for NCs and PLTs in the matrix compared with the starting concentration in the bone marrow aspirate.

### Evaluation of osteogenesis in TEB fabricated by PLL-DBM enriched bone marrow cells in goat intertransverse fusion model

#### Graft materials

The following four groups of graft materials were evaluated: IA, TEB fabricated by PLL-DBM-enriched bone marrow; IB, autogenous iliac bone; IIC, TEB fabricated by DBM-enriched bone marrow; IID, blank DBM.

#### TEB fabricated by PLL-DBM and DBM intraoperatively enriched bone marrow cells

PLL-DBM material (5 g) was tidily arranged in the filter bowl of the CELLECT device. Bone marrow (15 ml) was harvested from the left and right ilia, respectively, according to the method of Muschler *et al* (8), then 30 ml bone marrow was injected into the filter bowl of the CELLECT device and slowly flowed through the PLL-DBM material under the negative pressure pumping role of the CELLECT device for up to three circulations. Bone marrow stem cells and growth factors adhered to the bone matrix, and then the TEB (graft materials of group IA) were fabricated. DBM material (5 g) was arranged in the filter bowl of the CELLECT device and, according to the same method, the TEB (graft materials of group IIC) were fabricated.

#### Goat intertransverse fusion model

Twenty healthy adult male goats, 6–8 months old, 22–25 kg (average 23.8 kg), were offered by the Animal Center of the General Hospital of the Armed Police Force of Guangxi, and the animal experiments were approved by the Ethics Committee of Guangxi (Nanning, China). The 20 goats were randomly divided into two groups (I and II) with 10 goats in each group. The bilateral L3/4 vertebral lamina and transverse processes of the goats were exposed and the bone cortices were removed to prepare the bone beds in all goats. The graft materials of the IA and IB groups were implanted respectively in the left and right transverse process bone beds of L3/4 of group I goats, while the graft materials of the IIC and IID groups were implanted respectively in the left and right transverse process bone beds of L3/4 of group II goats. The fusion site included the gap between the transverse processes and the space between the lamina at each site, and each site required 5 g graft materials. The graft materials in the four groups (IA, IB, IIC and IID) were equal and Luque rods (Shanghai Medical Instruments, Inc., Shanghai, China) were used for posterior fixture. The goats received intramuscular injections of 800,000 units per injection, twice a day following surgery. The activities, eating and wound healing of the animals were observed post-operatively.

### Detection index

#### Radiographic analysis

All goats from groups I and II were sacrificed at 16 weeks after surgery. The lumbar spine was harvested intact, removing the internal fixators and soft tissues. Radiographs of the lumbar spine were captured using a DirectView CR900 device (Kodak Inc., Rochester, NY, USA). X-ray exposure was maintained at a constant for all animals at 70 kV for 3.2 mAs.

#### Computed tomography (CT)

Quantitative assessment of the bone formation in each fusion segment was conducted using a three-dimensional CT scanner (Siemens Medical Systems Inc., Erlangen, Germany) to determine the CT value. Scanning was performed at 125 kV(p), 220 mA, 1 sec helical mode and 2 mm collimation. Images were reconstructed using a bone algorithm and an image-to-image overlap at a slice thickness of 1 mm. Original software (D-image Goat 2 for Unix system; Santa Cruz Operation, Santa Cruz, CA, USA) was used to calculate the CT value, and the scanning area for the CT value was defined by the *de novo* bone between the transverse processes.

#### Histological observation

Decalcified samples were embedded in paraffin. Sagittal sections were performed along the fusion sites and through the transverse processes, and stained with hematoxylin and eosin.

#### Mechanical testing

Mechanical testing was conducted using an RGT Cybernation Materials Testing system (Shenzen Reger Instrument Co., Ltd., Shenzhen, China), and the data on maximum load and bending strength were obtained using a custom three-point bending device.

### Statistical analysis

The SPSS 11.0 statistical software package (SPSS Inc., Chicago, IL, USA) was used for analysis, and all measured data are presented as the mean ± standard deviation. The Student’s t-test was used for comparisons between two groups and variance analysis was used for comparisons among groups, with P<0.05 indicating statistical significance.

## Results

### Scanning electron microscopy observations

The PLL-DBM materials had a natural three-dimensional mesh structure, a high porosity and a high connectivity rate of interspaces. The aperture of the PLL-DBM (n=10) was 472.5l±7.02 μm and the porosity rate was 78.15±6.45%. However, the aperture of the DBM (n=10) was 478.5l±8.03 μm and porosity rate was 80.25±7.46%. Therefore, the apertures and porosity rates exhibited no significant differences between the two materials (P>0.05). The PLL-DBM surface and inner wall of mesh were covered by a milky white PLL coat, and the PLL formed a spider web-like mesh structure in the interspaces (Fig. 1).

### Infrared spectrum analysis

The C-O stretching vibration peak of the amide contained in PLL was at 1,657 cm^−1^, and the phosphate stretching vibration peak of the phosphoric acid in DBM was at 1,034 cm^−1^. The vibration peak of PLL-DBM increased at 1,657 cm^−1^ enhancement and did not change at 1,034 cm^−1^ (Fig. 2).

### Enrichment effect of PLL-DBM for NCs and PLTs

The α value for NCs and PLTs in PLL-DBM compared with the starting concentration in the original bone marrow was superior to that in DBM, and was significantly different (P<0.01) (Table I).

### Osteogenic ability observations

#### General observations

Following the surgery, one goat had an incision infection that healed subsequent to removing the sutures, draining and administration of antibiotic treatment. The remaining goats survived without incident. Subsequent to the goats being sacrificed and the internal fixators and soft tissues being removed, it was revealed that in 2/10 goats in group I, the bone fusion of IA grafts was worse than that of IB grafts, while the remaining eight goats showed similar osteogenic abilities between the IA and IB grafts, with complete fusion in all. In group II, it was observed in all goats that the bone fusion of IIC grafts was improved compared with that of IID grafts. The bone fusion of IA and IB grafts in group I was significantly improved compared with that of IIC and IID grafts in group II.

#### X-ray analysis

Sixteen weeks after the surgery, the fusion range of the IA and B groups was similar, with complete fusion in all, and the bone density was the same as that of the transverse processes (Fig. 3A). However, the fusion range of the IIC group was significantly lower than that of the IA and IB groups, and only the segment around the inner side of the vertebra had partly fused in the IIC group. No fusion was observed in the IID group; there were only island-like osteogenic chips between the transverse processes (Fig. 3B).

#### Three-dimensional CT analysis

Image reconstructions showed that the fusion range of the IA and IB groups was similar (Fig. 4), and a number of bones had formed outward along the vertebral lamina at the cross-section in the IA and IB groups and fused completely (Fig. 5). The CT value of the IA group was 696.76±102.75 Hounsfield unit (HU; n=10) and that of the IB group was 766.03±69.24 HU (n=10), thus showing no significant difference between the IA and B groups (P>0.05)*.* In the IIC group, only part-fusion was identified. The CT value was 488.63±76.40 HU (n=10), which was significantly lower than that in the IA and IB groups (P<0.01). In the IID group, where only small island-like bones had formed, the CT value was 91.83±31.87 HU (n=10), which was significantly lower when compared with that of the IA, IB and IIC groups (P<0.01) (Fig. 6).

#### Histological observations

The histological results showed that a number of woven bones had formed and that marrow-like tissue was present in the IA and IB groups. The osteoblasts around the graft were active; however, a number of fibrous tissues, which had not yet formed bone, could be observed in the center in the IIC group. A number of fibrous tissues and only a few small piece-like bones had formed in the IID group (Fig. 7).

#### Biomechanical testing

The maximum load and bending strength in the IA group exhibited no significant difference compared with those in the IB group (P>0.05). The values in the IA group were higher than those in the IIC group (P<0.01 and P<0.05, respectively), and those in the IB group were higher than those in the IIC group (both P<0.01). In addition, the values in the IIC group were significantly higher than those in the IID group (both P<0.01) (Table II).

## Discussion

The purpose of this study was to improve the adhesion effect of matrix materials used in SCR technology for bone marrow cells by using PLL to modify the surface and pore wall of DBM. Furthermore, the study aimed to improve the osteogenic potential of the matrix material, to provide an ideal matrix material for the SCR technology and to verify the osteogenic potential of the matrix material PLL-DBM in the goat transverse process model in order to provide an experimental basis for clinical applications.

The results of this study showed that PLL-DBM, which was DBM modified by PLL, was an ideal enriched matrix. Scanning electron microscope and infrared spectrum analyses showed that PLL combined well with DBM. Scanned with an electron microscope, PLL-DBM had a natural three-dimensional mesh structure, with an average micropore diameter of 472.5l±7.02 μm and a porosity rate of 78.15±6.45%. These values were consistent with the parameters of an ideal bone tissue engineering scaffold material (20). The PLL-DBM surface and inner wall of mesh were covered by a milky white PLL coat, and PLL formed a spider web-like mesh structure in the interspaces, which provided a physical space structure for the adhesion of seed cells. This not only facilitated the adhesion of seed cells but also facilitated the formation of new bones. The enrichment effect of PLL-DBM for bone marrow NCs and PLTs was significantly superior to that of pure DBM (P<0.01). The osteogenesis in the goat spinal transverse processes, X-ray samples and three-dimensional CT showed that the fusion range of the TEB fabricated by PLL-DBM-enriched bone marrow group, which was similar to that of autologous iliac bone, was markedly superior to that of the TEB fabricated by DBM-enriched bone marrow group and the blank DBM group. The TEB fabricated by PLL-DBM-enriched bone marrow group had a CT value that exhibited no significant difference from that of autologous iliac bone (P>0.05) and was also significantly higher than that of the TEB fabricated by DBM-enriched bone marrow and blank DBM groups (P<0.01). These results were consistent with those of the histological and biomechanical performance. The results showed that the TEB fabricated by PLL-DBM-enriched bone marrow not only exhibited an improved enrichment effect for bone marrow cells, but also showed an osteogenic ability that was similar to that of the autologous iliac bone and better than that of the TEB fabricated by DBM-enriched bone marrow.

Muschler *et al* (10,11) successively selected allograft cancellous chips and demineralized cortical bone powder as matrices and applied SCR technology to enrich bone marrow cells, the results showing that connective tissue progenitors in the matrix material increased significantly. This material was then mixed with non-heparinized bone marrow clots, and the score and fusion range of the mixture were significantly improved compared with those in other control groups in the canine spinal posterior vertebral lamina fusion model. However, the material’s enrichment effect for NCs was 2.7-fold, which was significantly lower than the results of this study (5.06-fold); this was mainly due to the matrix material having not been modified by an adhesion agent. Improving the adhesion property of enriched matrix for bone marrow to increase the number of cells that are capable of promoting osteogenesis in the matrix is at the core of SCR technology. Therefore in the present study, the PLL-DBM, in which PLL was used to modify the surface and pore wall of DBM, had an important application value.

PLL is a multivalent cation polymer formed by the lysine monomer. PLL is polymerized by a number of amino acid fragments through covalent bonds and van der Waals forces, and can be decomposed into lysine following metabolization in the human body without any side effects (21). PLL was previously used as an adhibiting agent in immunohistochemistry tests (22). However, the use of PLL as a surface modifier of enriched matrices has not been previously reported, to the best of our knowledge. The results of the present study showed that PLL was a good surface modifier of matrix material. The reasons for this may be that: i) Lysine residues fixed on the surface of the material with a positive charge could enhance the adhesion effect for cells with a negative charge (23); ii) the amidogens of PLL bound with proteoglycans on the cells’ surface and promoted the adhesion effect for cells (24); or iii) the micropore mesh structure in the pores of DBM enhanced the surface area, which was conducive to selecting a certain size of cell to adhere.

In theory, the four groups of graft materials, IA, IB, IIC and IID, should be designed using the same individual animals in order to reduce differences between groups; however, the amount of bone marrow that each animal could provide had to be considered during grouping design. Previous experiments showed that only ~30 ml bone marrow, which was insufficient for the amount of bone marrow required in the IA and IIC groups (the amount of bone marrow required in each group was ~30 ml), could be harvested from the bilateral iliac bones of each goat (25). While bone marrow was not required in the IB and IID groups, the optimum design of this study was that 20 goats were divided into two groups (I and II), and the materials in the IA and IB groups were implanted into the gaps of the left and right L3/4 transverse processes of the individuals in group I, respectively, while the materials in the IIC and IID groups were implanted into the gaps of the left and right L3/4 transverse processes of the individuals in group II. Thus, not only could the amount of bone marrow be guaranteed and the number of required animals reduced, but the differences between the groups could be minimized.

There are a few mesenchymal stem cells or osteoblast precursor cells in bone marrow (26), although it is difficult to use SCR technology to enhance the number of stem cells to the magnitude of mesenchymal stem cells inoculated by TEB conventionally fabricated by cell proliferation *in vitro*. In the SCR process, certain osteogenic factors in bone marrow, including PLT-derived growth factor (PDGF) and transforming growth factor-β (TGF-β), are also adhered and enriched at the same time, and these factors can promote the proliferation of stem cells and osteogenic differentiation in the body. In addition, other stem cells in enriched bone marrow, including hematopoietic stem cells, exert a synergistic effect by promoting the vascularization of bone repair materials (19). The bone marrow NCs detected in this experiment included not only mesenchymal stem cells, which had an osteogenic activity, but also hematopoietic stem cells. Mesenchymal stem cells themselves also contributed to the secretion of OIFs and collected OIFs from implanted receptors through chemotaxis in the body. Furthermore, PLTs could release OIFs such as PDGF and TGF-β. Therefore, not only cells in the matrix, but also the factors enriched by the matrix and OIFs secreted by enriched cells, play an important role in osteogenesis in SCR technology. This study detected the enrichment effects of PLL-DBM scaffold material for bone marrow NC and PLT concentration through SCR technology, which could reflect indirectly the adhesion and enrichment effects of the material for the effective osteogenic components. In addition, an automatic blood cell analyzer could be applied simply without cell culture *in vitro* and was convenient for the initial screening of a large number of materials.

The limitations of this study include the fact that animals were mainly used as the experimental specimens, so the osteogenic effect of the TEB fabricated in this study requires further clinical trials in the human body. In addition, only the enrichment effects of NCs and PLTs were detected in this experiment. The bone growth factors in the matrix materials were not detected and require verification in further experiments.

In conclusion, SCR technology in which PLL-DBM is used as an enriched matrix could successfully enrich the effective osteogenic components in bone marrow. TEB with high osteogenic activity could be fabricated rapidly during the procedure and used as a bone graft material to promote spinal fusion. The results were positive in the animal experiment and the osteogenic potential was similar to that of autologous ilium. PLL-DBM material is convenient to store and transport, and can be used at any time. SCR technology is safe, fast and inexpensive, and does not require cell culture *in vitro*. The effective osteogenic components of bone marrow increased following enrichment and the osteogenic effect was evident, indicating that SCR technology with a PLL-DBM enriched matrix may have a relatively wide clinical potential.

## Figures and Tables

**Figure 1:** Electron microscope images of (A) DBM and (B) PLL-DBM. The PLL-DBM surface and inner wall of mesh were covered by a milky white PLL coat, and the PLL formed a spider web-like mesh structure in the interspaces. DBM, demineralized bone matrix; PLL-DBM, DBM coated with poly-L-lysine.

**Figure 2:** PLL-DBM infrared spectrum: The characteristic peak of PLL-DBM was at 1,657 cm^−1^ and the enhanced peaks occurred where PLL vibration peaks were identified, indicating that PLL combines well with DBM. PLL, poly-L-lysine; DBM, demineralized bone matrix; PLL-DBM, DBM coated with PLL.

**Figure 3:** X-Ray images of samples in groups (frontal view). (A) The bones fused well in the IA and IB groups; (B) only a section around the inner side of the vertebra fused in the IIC group and no fusion was identified in the IID group.

**Figure 4:** Image reconstructions (rear view). (A) The bones fused well in the IA and IB groups; (B) part-fusion of bones was observed in the IIC group and only small groups of island-like bones were formed in the IID group.

**Figure 5:** Three-dimensional computed tomography (cross-section). (A) A number of bones were formed outward along the vertebral lamina at the cross-section in the IA and IB groups; (B) only a few bones formed outward in the IIC group and no bones formed outward in the IID group.

**Figure 6:** Comparison of CT values for all groups: ^a^P<0.01 vs. the IA group; ^b^P<0.01 vs. the IB group; ^c^P<0.01vs. the IIC group. CT, computed tomography.

**Figure 7:** Histological micrographs (hematoxylin and eosin staining; magnification, ×40). A number of woven bones (Q) had formed and marrow-like tissue (→) was observed in the (A) IA and (B) IB groups; (C) ossification around the graft was active (→), but a number of fibrous tissues (β), which had not yet formed bone, were observed in the center in the IIC group; (D) fibrous tissue (β) was the predominant feature in the IID group, with only a few small, piece-like bones.

**Table I:** Statistical results of fold increase in concentration relative to the starting concentration for NCs and PLTs.

Group	NCs	PLTs
DBM	1.60±0.37	2.18±0.42
PLL-DBM	5.06±0.60^a^	5.68±0.50^a^

Data (n=12) are presented as the mean ± standard deviation.

a P<0.01 vs. the DBM group.

NC, nucleated cell; PLT, platelet; DBM, demineralized bone matrix; PLL-DBM, DBM coated with poly-L-lysine.

**Table II:** Comparison of biomechanical performances.

Group	Maximum load (N)	Bending strength (MPa)
IA	72.29±16.62	19.15±3.88
IB	77.89±14.26	21.19±3.79
IIC	53.89±17.32^a^,^b^	14.36±2.89^b^,^c^
IID	15.43±5.77^a^,^b^,^d^	6.52±3.03^a^,^b^,^d^

Data (n=10) are presented as mean ± standard deviation.

a P<0.01 vs. the IA group;

b P<0.01 vs. the IB group;

c P<0.05 vs. the IA group;

d P<0.01 vs. the IIC group.
